The article "A Scoring Model Based on Neutrophil to Lymphocyte Ratio Predicts Recurrence of HBV-Associated Hepatocellular Carcinoma after Liver Transplantation" was retracted in 2019. Reasons: lack of ethics approval or compliance; missing or withdrawn patient consent; ethical violations by an author.

# A Scoring Model Based on Neutrophil to Lymphocyte Ratio Predicts Recurrence of HBV-Associated Hepatocellular Carcinoma after Liver Transplantation

**DOI:** 10.1371/journal.pone.0025295

**Published:** 2011-09-26

**Authors:** Guo-Ying Wang, Yang Yang, Hua Li, Jian Zhang, Nan Jiang, Min-Ru Li, Huan-Bing Zhu, Qi Zhang, Gui-Hua Chen

**Affiliations:** 1 Liver Transplantation Center, Third Affiliated Hospital, Sun Yat-sen University, Guangzhou, Guangdong, China; 2 Guangdong Provincial Key Laboratory of Liver Disease Research, Guangzhou, Guangdong, China; The University of Hong Kong, China

## Abstract

**Background:**

Neutrophil to lymphocyte ratio (NLR) has been proposed to predict prognosis of hepatocellular carcinoma (HCC). However, the cut-off values are empirical. We determined the optimal cut-off value to predict HCC recurrence after liver transplantation (LT) and further established a scoring model based on NLR.

**Methodology/Principal Findings:**

We analyzed the outcome of 101 HBV-associated HCC patients undergoing LT. Preoperative risk factors for tumor recurrence were evaluated by univariate analysis. By using ROC analysis, NLR≥3 was considered elevated. The disease-free survival (DFS) and overall survival (OS) for patients with high NLR was significantly worse than that for patients with normal NLR (the 5-year DFS and OS of 28.5% and 19.5% vs. 64.9% and 61.8%, respectively; *P*<0.001). Univariate analysis revealed that tumor size >5 cm, tumor number >3, macrovascular invasion, AFP≥400 µg/L, NLR≥3, and HBV-DNA level >5 log10 copies/mL were preoperative predictors of DFS. Cox regression analysis showed macrovascular invasion, tumor number, and high NLR were independent prognostic factors. We then established a preoperative prognostic score based on multivariate analysis. Each factor was given a score of 1. Area under the ROC curve of the score was 0.781. All nine patients with score 3 developed recurrence within 6 months after LT. Of 71 patients without vascular invasion, three patients with both tumor number >3 and NLR≥3 developed recurrence within 14 months after LT while the 5-year DFS and OS for patients with a score of 0 or 1 were 68.1% and 62.8%, respectively.

**Conclusions/Significance:**

Preoperative elevated NLR significantly increases the risk of recurrence in patients underwent LT for HCC. Patients with both NLR≥3 and tumor number >3 are not a good indication for LT. Our score model may aid in the selection of patients that would most benefit from transplantation for HCC.

## Introduction

Hepatocellular carcinoma (HCC) is one of the most prevalent cancers in the world, particularly in China. Chronic hepatitis B virus (HBV) infection is the leading risk factor for HCC in China. Liver transplantation (LT) appears to be an ideal treatment for unresectable HCC, which accounts for about 40% of the indications for LT in China [1]. In the absence of metastases and macroscopic vascular invasion, LT is the best available curative treatment option for patients with HCC on cirrhosis, since it not only removes the tumor completely but also effectively treats the underlying liver disease. However, before the introduction of Milan criteria in 1996 (single nodule ≤5 cm or two to three nodules ≤3 cm) [2], survival after transplantation was disappointing due to high rate of HCC recurrence. Milan criteria have significantly improved the outcome of LT for HCC and have been adopted by the United Network for Organ Sharing (UNOS) to guide patient selection. Many transplant centers confirmed the prognostic value of Milan criteria and established LT as therapy for HCC patients with cirrhosis [3]–[6]. However, the favorable outcomes have raised the question of whether selection criteria should be expanded. Over the last 10 years, expanded criteria have been most thoroughly investigated in an attempt to select suitable candidates beyond Milan criteria [3], [4], [7]–[9]. However, both Milan and the University of California San Francisco (UCSF) criteria (single nodule ≤6.5 cm, or two to three nodules with the largest nodule ≤4.5 cm and the total tumor burden ≤8 cm) solely rely on preoperative imaging findings including tumor number, size, and macrovascular invasion. Unfortunately, inaccuracy of radiological imaging remains a problem, particularly in cirrhosis [10]. Furthermore, radiological imaging can not detect microvascular invasion which has been associated with an increased risk of tumor recurrence. Although tumor size is a surrogate parameter for vascular invasion and poor differentiation [11], there are at least two reasons to explain why about 20% of patients who meet Milan criteria still develop tumor recurrence after LT. The first one is the inadequacy of preoperative imaging studies in assessing vascular invasion and tumor grade. Second, a proportion of patients tend to have some types of tumors which are more aggressive than others although the size of tumor was small. In addition, a proportion of patients with large tumors can achieved excellent outcomes after LT. Therefore, to identify the risk factors for recurrence is very important to limit or expand the indications for LT.

The article "A Scoring Model Based on Neutrophil to Lymphocyte Ratio Predicts Recurrence of HBV-Associated Hepatocellular Carcinoma after Liver Transplantation" was retracted in 2019. Reasons: lack of ethics approval or compliance; missing or withdrawn patient consent; ethical violations by an author.

Numerous clinical and experimental data have widely developed the concept that inflammation is a critical component of tumor progression [12], [13]. It is now accepted that the tumor microenvironment contributions to the development of angiogenesis. Several inflammatory markers such as C reactive protein have been suggested as surrogate markers for HCC [14]. One such a simple and effective marker of inflammation that has been linked with several gastroenterological malignancies is the neutrophil-lymphocyte ratio (NLR). An elevated NLR has been shown to be an indictor of poor outcome in patients undergoing hepatic resection for colorectal liver metastasis [15], [16], and curative resection for HCC [17]. More recently, two studies have demonstrated the efficacy of the NLR in predicting outcome in patients undergoing LT for HCC [18], [19]. Elevated NLR significantly increases the risk for tumor recurrence after LT. However, in above all these studies, the cut-off value for NLR of 5 has been set empirically. The number of patients in these studies who had NLR more than 5 was small.

The aim of this study was to determine the optimal cut-off value for preoperative NLR in HCC patients undergoing LT and evaluate whether the new cut-off point for NLR correlates with tumor recurrence. Furthermore, we established a simple preoperative prognostic score model that may aid in the selection of patients that would most benefit from transplantation for HCC.

## Methods

### Patient selection

One hundred and one HBV-associated HCC patients treated with LT in our hospital (Third Affiliated Hospital, Sun Yat-sen University, Guangdong, China) during the 6-year period from October 2003 to June 2009 were enrolled in this study. Demographic, clinical, and laboratory data, including patient age, gender, white cell and differential counts within 7 days before surgery, serum alpha-fetoprotein (AFP) level, preoperative imaging data based on abdominal computed tomography or magnetic resonance imaging (tumor size, number, and macrovascular invasion), the history of pretransplant tumor therapy, HBV infection, HBV-DNA level, and explant pathology were recorded. Pretransplant tumor therapies included radiofrequency ablation, liver resection, ethanol ablation, transarterial chemoembolization, local radiotherapy and systemic chemotherapy. NLR was defined as the absolute neutrophil count divided by the absolute lymphocyte count. Final diagnosis of HCC was made by pathological examination of the explanted liver. The eligibility criteria for the patients studied are as follows: (a) all patients were HBV infected and none of them were hepatitis C virus-positive; (b) all patients were adults (more than 18 years of age); (c) complete clinical and laboratory data such as AFP level, tumor size, and tumor number were available. (d) any patients missing blood results within 7 days before surgery or missing preoperative imaging data within 1 month before surgery were excluded; (e) any patients demonstrating signs of preoperative sepsis were excluded; (f) none of the patients occurred gastrointestinal hemorrhage, undergoing pretransplant tumor therapy, or given hematopoietic agents such as G-CSF within 1 month before surgery as these conditions can result in a falsely elevated NLR; (g) any patients on high-dose steroids before transplantation were excluded; and (h) patients had no HCC on pathology or no any follow-up data were also excluded. This study was approved by the Institutional Review Board of Key Lab of Liver Disease Research in Guangdong Province. Informed written consent was obtained according to the Declaration of Helsinki.

The article "A Scoring Model Based on Neutrophil to Lymphocyte Ratio Predicts Recurrence of HBV-Associated Hepatocellular Carcinoma after Liver Transplantation" was retracted in 2019. Reasons: lack of ethics approval or compliance; missing or withdrawn patient consent; ethical violations by an author.

### Surgery and postoperative management

Liver transplants are performed using standard techniques without the use of venovenous bypass. The piggyback's technique with suprahepatic venacavaplasty of retrohepatic cava extention for LT was performed in most patients. Generally, our transplant center's postoperative immunosuppression regimen consisted of calcineurin inhibitors and steroids. Steroids were discontinued within 3 months.

### Follow-up

After LT, patients were regularly followed up at the outpatient clinics. Abdominal and chest CT were monitored every 3 months in the first two postoperative years, followed by every 6 months in the third year. AFP measurement is performed every month in the first year and then every 3 months for the next two years. In the following years, an annual abdominal CT scan was performed. CT or MR imaging of the abdomen pelvis, chest and bone scan was monitored to define suspicious lesions demonstrated on CT or raised AFP level.

### Statistical analysis

SPSS for Windows program (version 13.0) and MedCalc statistical software v11.3.0.0 were used to analyze the data. Patients were censored at last follow-up if still alive or lost to follow-up. A suitable cut-off value for elevated NLR was selected using the receiver operating characteristic (ROC) curve analysis. The independent samples *t* test, and Pearson's chi-square (χ^2^) test were used to analyze differences in clinicopathological features between patients with high and normal NLR. The clinicopathologic factors that were significant differences between patients with high and normal NLR were entered into a stepwise forward logistic regression model to determine their independent risk factors. Survival curves were determined by the Kaplan–Meier method. Potential predictors of patient outcomes and disease-free survival were entered into univariate Kaplan–Meier models and tested by the log-rank statistic. Preoperative clinicopathologic factors that had significant impact on disease-free survival in the univariate analysis were entered into a multivariate Cox regression model (stepwise forward method) to determine their independent effect. A preoperative prognostic score model was established to predict tumor recurrence based on preoperative factors that were significant on multivariate analysis. Univariate Cox proportional hazards regression analysis was applied to estimate the hazard ratio for the risk of tumor recurrence. By using MedCalc statistical software, the area under the ROC curve (AUC) for the score model was measured and then compared with the Milan, UCSF, and HangZhou criteria (tumor <8 cm, or ≥8 cm but with well differentiation and serum AFP≤400 ng/mL) [20]. Variables with *P*<0.05 were considered statistically significant.

The article "A Scoring Model Based on Neutrophil to Lymphocyte Ratio Predicts Recurrence of HBV-Associated Hepatocellular Carcinoma after Liver Transplantation" was retracted in 2019. Reasons: lack of ethics approval or compliance; missing or withdrawn patient consent; ethical violations by an author.

## Results

### Patient demographics and outcomes

Ninety-two patients (91.1%) were men and 9 (8.9%) women. The mean age of patients at transplant was 48.4 years (range: 27–72 years). Thirty-five patients (34.7%) received pretransplant tumor therapy. Fifty-one patients died during follow-up and 4 died within one month post-transplantation. Of 42 patients (41.2%) developed tumor recurrence, 28 (66.7%) developed recurrence within 1 year and 38 (90.5%) developed recurrence within 2 years after LT. Mean follow-up time was 2.85 years (range: 0.38–6.22 years) with 7 patients lost to follow-up. The 1-, 3-, and 5-year (yr) overall survival (OS) and disease-free survival (DFS) rates for all patients included in this study were 80.2%, 55.4%, and 47.6% and 70.7%, 55.6%, and 53.6%, respectively (Figure S1).

### An optimal cut-off value for elevated NLR

By using ROC curve analysis, we determined the optimal cut-off value for elevated NLR. The area under the receiver operating characteristic curves was 0.667 with a 95% confidence interval (95% CI) for the area being between 0.557 and 0.777 (Figure S2). A cut-off value of 2.48 presented a sensitivity of 59.5% and a specificity of 71.2%. When the cut-off point was increased to 2.99, the sensitivity was 50% and the specificity was 79.7%. Therefore, the cut-off value of 3.0 was used in this study.

### Risk factors for recurrence of hepatocellular carcinoma after LT

Univariate analysis of factors affecting disease-free survival was shown in Table 1. More than three tumor nodules, size of largest tumor >5 cm, macrovascular invasion, AFP ≥400 ng/mL, NLR≥3, and HBV-DNA level >5 log10 copies/mL were all preoperative prognostic predictors of poorer DFS. The NLR was elevated at ≥3 in 34 patients (33.3%). A significant difference in DFS existed between patients with normal and elevated NLR. The 5-yr DFS of 64.9% in patients with a normal NLR compared with 28.5% in patients with an elevated NLR, respectively, *P*<0.001, Figure 1A). Of 30 patients with macrovascular invasion, 3 died within 1 month after transplantation; 2 died from biliary infection and multiple organ dysfunction syndrome 5 and 7 months after transplantation, respectively; 4 had no tumor recurrence during 5 years of follow-up; tumor recurrence were detected in all the other 21 patients during 18 months of follow-up. Of 4 patients without tumor recurrence, 3 had no macroscopic tumor thrombus in the explant liver and histopathologic analysis revealed no evidence of microvascular invasion. Of 71 patients without macrovascular invasion on preoperative imaging, 16 patients with high NLR had slightly lower DFS than patients with normal NLR but no statistically significant difference was found (5-yr DFS of 70.8% vs. 53.0%, respectively, *P* = 0.106, Figure S3A).

The article "A Scoring Model Based on Neutrophil to Lymphocyte Ratio Predicts Recurrence of HBV-Associated Hepatocellular Carcinoma after Liver Transplantation" was retracted in 2019. Reasons: lack of ethics approval or compliance; missing or withdrawn patient consent; ethical violations by an author.

**Figure 1:** Kaplan-Meier survival curves for patients with high or normal NLR. There was a significant difference in DFS and OS between patients with low and high NLR. The 5-yr DFS (A) and OS (B) for patients with normal or high NLR were 64.9%, 28.5%, and 61.8%, 19.5%, respectively (both *P*<0.001).

**Table 1:** Preoperative factors affecting disease-free survival and overall survival.

Category	Subcategory (n)	Disease-free survival				Overall survival			
		5 years	Univariate analysis	Multivariate analysis	HR (95%CI)	5 years	Univariate analysis	Multivariate analysis	HR (95%CI)
Gender	Male (92)	52.0%	0.271	–		46.4%	0.360	–	
	Female (9)	72.9%				58.3%			
Age	<60 years (87)	72.9%	0.189	–		46.7%	0.703	–	
	≥60 years (14)	63.5%				50.0%			
Preoperative tumor therapy	Yes (35)	63.5%	0.189	–		42.2%	0.171	–	
	No (66)	47.9%				57.8%			
Size of largest tumor	≤3 cm (26)	69.9%	0.002	NS		66.7%	<0.001	NS	
	≤5 cm (34)	61.5%				62.8%			
	≤8 cm (14)	40.8%				27.8%			
	>8 cm (27)	31.1%				20.0%			
Tumor numbers	≤3 (68)	67.9%	<0.001	<0.001	4.117 (2.087–8.123)	58.0%	<0.001	<0.001	3.013 (1.644–5.524)
	>3 (33)	24.5%				26.4%			
Vascular invasion	No (71)	66.8%	<0.001	<0.001	3.908 (1.965–7.772)	61.6%	<0.001	<0.001	3.253 (1.734–7.772)
	Yes (30)	17.2%				15.0%			
AFP	<400 ng/mL (61)	65.9%	<0.001	NS		62.6%	<0.001	NS	
	≥400 ng/mL (40)	32.1%				24.6%			
NLR	<3 (68)	64.9%	<0.001	<0.001	3.665 (1.799–7.466)	61.8%	<0.001	<0.001	2.654 (1.419–4.964)
	≥3 (33)	28.5%				19.5%			
HBV-DNA level >5 log10 copies/mL	No (88)	60.8%	0.016	NS		51.9%	0.021	NS	
	Yes (13)	10.4%				19.2%			

Abbreviation: CI, confidence interval; HR, hazard ratio; NS, not significant.

Multivariate regression analysis was performed on all 6 preoperative factors that were statistically significant difference in DFS by univariate analysis. The results revealed that the presence of macrovascular invasion, tumor number >3, NLR ≥3 were the independent prognostic predictors of poor DFS (Table 1).

The article "A Scoring Model Based on Neutrophil to Lymphocyte Ratio Predicts Recurrence of HBV-Associated Hepatocellular Carcinoma after Liver Transplantation" was retracted in 2019. Reasons: lack of ethics approval or compliance; missing or withdrawn patient consent; ethical violations by an author.

With regards to overall survival, there was a significant difference in overall survival between patients with low and high NLR (5-yr OS of 61.8% vs. 19.5%, respectively, *P*<0.001, Figure 1B). Again, on multivariate analysis, the presence of macrovascular invasion, tumor number >3, NLR≥3 were the independent prognostic predictors of overall survival (Table 1). Of patients without macrovascular invasion, patients with high NLR had significant lower OS than patients with normal NLR (5-yr OS of 69.6% vs. 36.7%, respectively, *P* = 0.037, Figure S3B).

### The analysis of clinicopathologic characters in patients with elevated NLR

The analysis of clinicopathologic characters in patients with normal or elevated NLR is shown in Table 2. Size of largest tumor >5 cm, macrovascular invasion, AFP≥400 ng/mL, outside Milan, outside UCSF, and outside HangZhou criteria were significant differences between patients with normal and high NLR based on univariate analysis. Furthermore, multivariate logistic regression analysis using all three parameters, eg, size of largest tumor, macrovascular invasion, and AFP, revealed that only macrovascular invasion remained associated with high NLR (*P* = 0.001, relative risk = 4.495, 95% CI = 1.086–11.188).

**Table 2:** Comparison of clinicopathological features of patients with elevated and normal NLR.

Factors	NLR<3 (n = 68)	NLR≥3 (n = 33)	*t* or χ^2^	*P*
Age (mean)	48.8 years	47.5 years	0.62	0.536
Male	61 (89.7%)	31 (93.9%)	0.108	0.743
Preoperative tumor therapy	27 (39.7%)	8 (24.2%)	2.346	0.126
Size of largest tumor >5 cm	21 (30.9%)	20 (60.6%)	8.140	0.004
Tumor numbers >3	21 (30.9%)	12 (36.4%)	0.303	0.582
Vascular invasion	13 (19.1%)	17 (51.5%)	11.168	0.001
AFP≥400 ng/mL	20 (29.4%)	20 (60.6%)	9.039	0.003
HBV-DNA level >5 log10 copies/mL	9 (13.2%)	4 (12.1%)	0.000	1.000
Outside Milan criteria	36 (52.9%)	29 (87.9%)	11.823	0.001
Outside UCSF criteria	31 (45.6%)	25 (75.6%)	8.186	0.004
Outside HangZhou criteria	18 (26.5%)	21 (63.6%)	12.947	<0.001

Abbreviation: NLR, neutrophil-lymphocyte ratio.

### Classification of patients according to NLR and the different criteria

In this study, 36 patients (35.6%) were within Milan criteria. Of the patients who were outside Milan, 9 and 26 were classified within UCSF and HangZhou criteria, respectively. The DFS of patients who were inside Milan criteria did not significantly differ from those patients outside Milan but within UCSF criteria (log rank test, *P* = 0.07), and similarly, patients outside Milan but within UCSF did not significantly differ from patients outside UCSF but within HangZhou criteria. However, patients within Milan had significantly better DFS than patients outside UCSF but within HangZhou criteria (log rank test, *P* = 0.001), and patients outside UCSF but within HangZhou criteria had significantly better DFS than patients outside HangZhou criteria (log rank test, *P* = 0.025), as shown in Figure 2A. Hangzhou criteria significantly expand the indications for liver transplantation with acceptable rates of 5-yr DFS and OS (70.3% and 65.3%, respectively, Figure S4).

The article "A Scoring Model Based on Neutrophil to Lymphocyte Ratio Predicts Recurrence of HBV-Associated Hepatocellular Carcinoma after Liver Transplantation" was retracted in 2019. Reasons: lack of ethics approval or compliance; missing or withdrawn patient consent; ethical violations by an author.

**Figure 2:** Disease-free survival for patients classified according to NLR and the different criteria. (A) The Kaplan-Meier curves for patients classified according to the Milan, UCSF and HangZhou criteria showed patients within Milan had significantly better DFS than patients outside UCSF but within HangZhou criteria (log rank test, *P* = 0.001). (B) Among patients beyond Milan criteria, a significant difference in DFS existed between patients with normal and elevated NLR (log rank test, *P* = 0.015).

Four patients who met Milan criteria had an elevated NLR. Of 32 patients with normal NLR and within Milan criteria, only three patients have shown tumor recurrence within 1 year and have died within 2 years after OLT. No tumor recurrence was found in all the other 29 patients during follow-up. There was no significant difference in DFS between patients with normal and high NLR of patients who met Milan criteria. However, of the patients beyond the criteria, a significant difference in DFS existed between patients with normal and elevated NLR; 29 patients with a high NLR having the 5-yr DFS of 21.5% compared with 42.2% in 36 patients with a normal NLR, respectively (*P* = 0.015, Figure 2B). The similar results were obtained when patients were reclassified according to UCSF and HangZhou criteria. Of 56 patients beyond UCSF criteria, 25 patients with a high NLR having a 5-yr DFS of 10.7% compared with 41.2% in 31 patients with a normal NLR (*P* = 0.001).

### A preoperative prognostic scoring model

Based on the preoperative recurrence score recently published by Halazun et al. [18] for tumor recurrence in patients transplanted for HCC, we established a preoperative prognostic score model, using the 3 preoperative prognostic factors found to be significant on multivariate analysis, namely, vascular invasion, tumor number, and NLR. Each factor was given a score of 1 and then patients were divided into 4 categories. Differences in DFS stratified according to the preoperative prognostic scores are shown in Figure 3A. The 5-yr DFS for 43 patients with a score of 0 was 81.9%, compared with 53.6% for 30 patients with a score of 1 (*P* = 0.018). The DFS in 19 patients with a score of 2 decreased sharply (the 1- and 2-yr survivals of 32.7% and 6.5%, respectively). Nine patients with a score of 3 had the worst DFS of all groups. All these patients showed tumor recurrence within 6 months and died within 17 months after LT. The median DFS for patients with a score of 2 and 3 were 3.8 and 8.5 months, respectively, compared with 5 years for patients with a score of 1. Patients with a score of 0 had minimal recurrence, with 36 patients (83.7%) being disease free at 5 years. Clearly, therefore, the DFS for patients with a score of 2 or 3 was significantly worse than that for patients with a score of 0 or 1 (the 1- and 3-yr DFS, 23.8% and 4.8% vs. 86.0% and 71.7%, respectively, *P*<0.001, Figure 3B).

The article "A Scoring Model Based on Neutrophil to Lymphocyte Ratio Predicts Recurrence of HBV-Associated Hepatocellular Carcinoma after Liver Transplantation" was retracted in 2019. Reasons: lack of ethics approval or compliance; missing or withdrawn patient consent; ethical violations by an author.

**Figure 3:** Disease-free survival for patients classified according to the preoperative prognostic score. (A) The Kaplan-Meier curves showed there was a significant difference in DFS among four groups of patients with score 0 to 3. (B) A significant difference in DFS existed when patients were reclassified into two groups (score 0 or 1, and 2 or 3).

Of 30 patients with macrovascular invasion on preoperative imaging, one of 3 patients with a score of 1 had no macroscopic tumor thrombus in the explant liver and histopathologic analysis revealed no evidence of microvascular invasion. He had no tumor recurrence during 23 months of follow-up. The other 27 patients had 2 or 3 scores. These results indicated that patients with a score of 2 or 3 were not a good indication for liver transplantation but patients with a score of 0 or 1 can achieve an acceptable survival after LT with a 5-yr DFS and OS of 69.1%, 63.8%, respectively.

The predictive value of the preoperative prognostic score model, as well as the value of Milan, UCSF and HangZhou criteria was assessed using univariate Cox proportional hazards regression analysis (Table 3). The preoperative prognostic score was superior to the Milan, UCSF and HangZhou criteria, with scores of 1, 2, and 3 having hazard ratios of 2.912, 15.533, and 48.715, respectively. ROC curve analysis of the preoperative prognostic score versus that of Milan, UCSF and HangZhou criteria is shown in Table 4 and Figure S5 by using MedCalc statistical software. The preoperative prognostic score was the most accurate at predicting recurrence with the AUC of 0.781 though no statistically significant difference was observed.

**Table 3:** Univariate Cox regression analysis of preoperative score model as well as Milan, UCSF and HangZhou criteria.

	*P*	Hazard Ratio	95% CI
Preoperative prognostic score = 0	—	—	—
Preoperative prognostic score = 1	0.023	2.912	1.161–7.305
Preoperative prognostic score = 2	<0.001	15.533	6.097–39.568
Preoperative prognostic score = 3	<0.001	48.715	13.974–169.825
Milan criteria	<0.001	8.528	3.035–23.960
UCSF criteria	<0.001	6.615	2.926–14.956
HangZhou criteria	<0.001	5.240	2.772–9.903

The article "A Scoring Model Based on Neutrophil to Lymphocyte Ratio Predicts Recurrence of HBV-Associated Hepatocellular Carcinoma after Liver Transplantation" was retracted in 2019. Reasons: lack of ethics approval or compliance; missing or withdrawn patient consent; ethical violations by an author.

**Table 4:** ROC curve analysis of preoperative prognostic score versus Milan, UCSF and HangZhou criteria.

	AUC	95% CI
Milan criteria	0.724	0.624–0.823
UCSF criteria	0.739	0.640–0.838
HangZhou criteria	0.699	0.593–0.806
Preoperative prognostic score	0.781	0.688–0.875

Abbreviation: AUC, the area under the ROC curve; CI, confidence interval; ROC, the receiver operating characteristic.

### Preoperative prognostic scores predict tumor recurrence in patients without macrovascular invasion

Because patients with gross vascular invasion of the portal vein, hepatic veins, or vena cava were not considered a good indication for LT due to the high rate of tumor recurrence, we next analyzed the prognostic value of our score model for patients without vascular invasion detected by preoperative imaging. Patients were divided into 3 categories. The results showed all 3 patients with a score of 2 got tumor recurrence within 14 months and died within 23 months after LT while the 5-yr DFS and OS for patients with a score of 0 and 1 were 81.4%, 74.2%, and 54.6%, 53.7%, respectively (Figure 4A and B). The DFS and OS for patients with a score of 2 was significantly worse than patients with a score of 1 (*P*<0.001 and  = 0.001, respectively). Of 26 patients with a score of 1, 13 patients with high NLR had slightly lower DFS rates than patients with more than 3 tumor nodules but no statistically significant difference was found (the 3- and 5-yr survivals, 68.4% and 45.6% vs. 76.9% and 59.8%, respectively, *P* = 0.756). Patients with scores of 1 and 2 had hazard ratios of 2.615 and 31.810, respectively. Patients with a score of 0 or 1 can achieve long-term survival after LT with a 5-yr DFS of 69.9% and OS of 64.4%, respectively. The preoperative prognostic score model for patients without vascular invasion revealed the strong associations of tumor recurrence risk with tumor numbers and high NLR with the AUC of 0.705 with the 95% CI of 0.565–0.844. These results indicated that patients without vascular invasion but with both elevated NLR and more than 3 tumor nodules were also not a good indication for LT. Our preoperative prognostic score significantly expand the indications for liver transplantation.

**Figure 4:** The prognostic value of the preoperative prognostic score model for patients without vascular invasion. The Kaplan-Meier curves showed there was a significant difference in DFS (A) and OS (B) between patients with a score of 2 and patients with a score of 0 or 1.

The article "A Scoring Model Based on Neutrophil to Lymphocyte Ratio Predicts Recurrence of HBV-Associated Hepatocellular Carcinoma after Liver Transplantation" was retracted in 2019. Reasons: lack of ethics approval or compliance; missing or withdrawn patient consent; ethical violations by an author.

## Discussion

Among appropriately selected candidates, LT for HCC provides excellent outcomes with 5-yr survival rates similar to patients undergoing LT for liver cirrhosis without HCC. However, about 20% of patients with Milan criteria still develop tumor recurrence after LT [2]. There remains controversy about expanding the criteria for selection of HCC patients for LT for a proportion of patients with tumor burden beyond Milan criteria may potentially benefit from LT. Lack of available liver donors is the main restricting factor for LT and contributes to prolonged waiting time, which is associated with increased drop out rates. However, expansion of selection criteria increases not only the risk of tumor recurrence, but also the need for donor organs, and further lengthens waiting time. Early experience demonstrated that tumor size was an important predictor of recurrence and survival for patients undergoing LT for HCC. But the preoperative tumor size can only be assessed by preoperative radiological imaging, which underestimates tumor stage in about 30% of cases, especially in patients with tumors beyond Milan criteria [8]. For all these reasons, there is an urgent need to develop new non-invasive biomarkers predicting patients at high risk of recurrence after hepatic resection or transplantation.

Consistent lines of evidence have suggested that there is a close relationship between the development of cancer and inflammation. Inflammation contributes to the development of at least 15% of all cancers, in particular, for the digestive system cancers [21]. Patients with HBV infections experience chronic inflammation which increases risk of liver cancer. Neutrophil to lymphocyte ratio (NLR), a simple and effective marker of inflammation, is easily calculated from routinely available data. During the past five years, some studies have demonstrated that an elevated NLR is an important prognostic factor in patients with a variety of digestive system malignancies including esophageal cancer [22], gastric cancer [23], [24], colorectal cancer [25], [26], colorectal liver metastases [15], [16], [27], pancreatic adenocarcinoma [28], intrahepatic cholangiocarcinoma [29], and HCC [17], [18]. However, in all these studies, the cut-off value for NLR of 5 has been set empirically except for one study of gastric cancer with the cut-off level of 4 based on Kaplan-Meier analysis. To our knowledge, this is the first report discussing the appropriate cut-off point of NLR in predicting prognosis in patients with HCC. First, we determined the optimal cut-off point for preoperative NLR to predict HCC patients with high risk of tumor recurrence after LT. By using ROC curve analysis, we found that the cut-off value of 3.0 had a relatively high specificity. Although patients with NLR values between 3.0 and 5.0 were classified as having an elevated NLR based on our new cut-off value, our results showed that patients with NLR<3 showed significantly better DFS and better OS than those of patients with NLR≥3. The results of multivariate regression analysis revealed that NLR≥3 was the independent prognostic predictor of poor DFS. This is consistent with the above studies. Although the relationship between elevated NLR and increased risk for early recurrence and poor prognosis is largely unclear, there are several possible mechanisms explaining the predictive role of preoperative elevated NLR. The systemic and local inflammatory response to tumor may provide a favorable environment for tumor invasion and metastases [13]. Furthermore, except for chronic inflammation caused by HBV and tumor itself, high expressions of granulocyte colony-stimulating factor in tumor tissue and macrophage colony-stimulating factor in peritumoral tissue are also associated with the elevated circulating neutrophils and poor prognosis [30]–[32]. Circulating elevated levels of vascular endothelial growth factor secreted mainly by circulating neutrophils have been associated with increased risk of recurrence in patients with HCC [33]. On the other hand, reduced lymphocyte infiltration, reflecting an impaired host immune response, has been shown to predict recurrence in HCC patients following LT [34]. NLR reflects an immune microenvironment that both favors tumor vascular invasion and suppresses the host immune surveillance. In addition, NLR can not only predict tumor recurrence but also be used for diagnosis of tumor. A recent study has showed that NLR can be a useful tool for preoperative diagnosis in patients with uterine sarcomas [35].

The article "A Scoring Model Based on Neutrophil to Lymphocyte Ratio Predicts Recurrence of HBV-Associated Hepatocellular Carcinoma after Liver Transplantation" was retracted in 2019. Reasons: lack of ethics approval or compliance; missing or withdrawn patient consent; ethical violations by an author.

Although univariate analysis in this study showed that tumor size, AFP level, and HBV-DNA level were preoperative prognostic predictors of poorer DFS, none of these factors were identified as independent predictors on multivariate analysis. However, this result did not mean that these factors were not associated with recurrence. In fact, previous studies have showed that tumor size >3 cm on imaging is an independent predictor of microvascular invasion [36], [37]. Our results showed a significant association between the elevated NLR and the tumor size, AFP level, and macrovascular invasion. Taken together, these results indicated that preoperative elevated NLR can indirectly reflect tumor burden, malignancy, invasion, and metastasis.

We found that more than 3 tumor nodules were an independent predictor of recurrence. The result was concomitant with some studies [37], [38] but not the others [20], [39], [40]. Multiple tumor nodules can be categorized into two types: multifocal occurrence and intrahepatic metastasis. HCC patient with intrahepatic metastasis has a poorer prognosis than those with multifocal occurrence. Although fast developed imaging techniques can detect small intrahepatic metastasis, we can not accurately distinguish intrahepatic metastasis from multifocal occurrence based on preoperative imaging. However, in our current study including 27 patients with tumor size >8 cm, we notified that multiple small satellite nodules seemed to surround a large main tumor. The different background of hepatitis may also partly explain that our results were different from that of other publications from Japan or Europe. HCC patients with HCV-associated cirrhosis have a higher incidence of multifocal occurrence than patients with HBV-related cirrhosis [41].

Based on multivariate analysis, we have therefore established a simple preoperative prognostic score model that is superior to the Milan, UCSF and HangZhou criteria at predicting recurrence, with an AUC of 0.781. All patients with a score of 3 showed tumor recurrence within 6 months after LT. The median DFS for patients with a score of 2 and 3 were 3.8 and 8.5 months, respectively. Clearly, LT for these patients is futile. As for patients without macrovascular invasion on radiological findings, all 3 patients with scores of 2 (both NLR≥3 and tumor nodules >3), who got recurrence within 14 months after LT, had hazard ratios of 31.810 with an AUC of 0.705. Whereas patients with a score of 0 or 1 may achieve similar survival outcomes as patients within HangZhou criteria, but including more patients (69 and 62 patients, respectively). These results indicated that patients without vascular invasion but with both elevated NLR and more than 3 tumor nodules were also not a good indication for LT. A similar study has demonstrated that a scoring model based on NLR before treatment offers a very informative method for predicting prognosis of gastric cancer [42].

Although we demonstrated the prognostic value of NLR in predicting recurrence, it would not be appropriate to conclude that LT should not be considered only because preoperative NLR is high. There are many other factors affecting NLR, such as an acute undetected infection, which affects the accuracy of prognostic prediction. In addition, all patients enrolled had a history of hepatitis B, which may bias the study since hepatitis C is the most common predisposing factor to HCC development in Western countries and Japan. In addition, our study was limited by the retrospective nature of the analysis and the relatively small number of patients was included in the report. Clearly, further prospective studies are needed to confirm and update our preoperative prognostic score model for the prediction of post-transplant tumor recurrence in patients with HCC.

The article "A Scoring Model Based on Neutrophil to Lymphocyte Ratio Predicts Recurrence of HBV-Associated Hepatocellular Carcinoma after Liver Transplantation" was retracted in 2019. Reasons: lack of ethics approval or compliance; missing or withdrawn patient consent; ethical violations by an author.

## Supporting Information

Figure S1 Disease-free survival (A) and overall survival (B) rates for all patients included in this study.
(TIF)

Figure S2 Receiver operating characteristic curve for NLR predicting tumor recurrence.
(TIF)

Figure S3 Kaplan-Meier survival curves for patients without macrovascular invasion and with high or normal NLR. Of patients without macrovascular invasion, the impact of high NLR on DFS was not statistically significant (A), but patients with high NLR had significant lower OS than patients with normal NLR (B).
(TIF)

Figure S4 Kaplan-Meier DFS (A) and OS (B) curves for patients with or beyond Hangzhou criteria.
(TIF)

Figure S5 Receiver operating characteristic curve for the different criteria predicting tumor recurrence.
(TIF)
